This article has been retracted.

# Knocking down ETS Proto-oncogene 1 (ETS1) alleviates the pyroptosis of renal tubular epithelial cells in patients with acute kidney injury by regulating the NLR family pyrin domain containing 3 (NLRP3) transcription

**DOI:** 10.1080/21655979.2022.2079242

**Published:** 2022-05-25

**Authors:** Chenxia Juan, Ye Zhu, Yan Chen, Yan Mao, Yan Zhou, Weiwei Zhu, Xufang Wang, Qian Wang

**Affiliations:** a Department of Nephrology, Jiangsu Province Hospital of Chinese Medicine, Affiliated Hospital of Nanjing University of Chinese Medicine, Nanjing, Jiangsu, China; b Department of Nephrology, Second Affiliated Hospital of Soochow University, Suzhou, Jiangsu, China; c Department of Nephrology, Jiangsu Province Geriatric Hospital, Jiangsu Province Official Hospital, Nanjing, Jiangsu, China; d Department of Pediatrics, the First Affiliated Hospital, Nanjing Medical University, Nanjing, Jiangsu, China; e Department of Pediatrics, Shanghai General Hospital, Shanghai Jiao Tong University School of Medicine, Songjiang, Shanghai, China

**Keywords:** acute kidney injury, ETS1, NLRP3, transcription, pyroptosis

## Abstract

Acute kidney injury (AKI) has a high mortality rate, but its pathogenesis remains unclear Lipopolysaccharide (LPS)-mediated renal tubular epithelial pyroptosis is involved in the pathogenesis of AKI. NLR family of pyrin domains containing 3 (NLRP3) plays an important role in pyroptosis. To further understand the transcriptional regulation mechanism of NLRP3, the peripheral blood of patients with AKI was analyzed in this study, showing that the levels of NLRP3 and cell pyroptosis in patients with AKI were significantly higher than those in normal controls. Furthermore, elevated levels of NLRP3 and cell pyroptosis were found in renal tubular epithelial cells after LPS treatment. Transcription factor ETS Proto-Oncogene 1 (ETS1) could bind to the upstream promoter transcription site of NLRP3 to transactivate NLRP3 in renal tubular epithelial cells. The cell pyroptosis level also decreased by knocking down ETS1. It is concluded that knocking down of ETS1 may reduce the renal tubular epithelial pyroptosis by regulating the transcription of NLRP3, thus relieving AKI. ETS1 is expected to be a molecular target for the treatment of AKI.

## Highlights

- NLRP3 is elevated in AKI patients and HK2 cells.
- ETS1 regulates NLRP3.
- ETS1 binds to NLRP3’s promoter.

## Introduction

Acute kidney injury (AKI) is a clinical condition that results in azotemia, electrolyte imbalances, and acid-base abnormalities. AKI is becoming increasingly common in hospitalized patients with poor long-term outcomes. For instance, the incidence of AKI in intensive care units is as high as 22–67% [1,2]. It is estimated that AKI in about half of the patients was attributed to severe sepsis with a mortality rate of 50–70% [3,4]. Although hemodynamic changes, inflammation, etc., have been proved to be linked to the sepsis-induced AKI [3], the pathophysiology of sepsis-induced AKI is still unknown.

AKI is characterized by damage to or death of renal tubular epithelial cells, and pyroptosis plays a key role in the pathogenesis of AKI [5]. The NLR family pyrin domain containing 3 (NLRP3) plays a vital role in pyroptosis, which has been defined as a pro-inflammatory programmed cell death pathway. NLRP3 inflammasome encoded by NLRP3 gene is an intracellular multi-protein complex involved in inflammatory response and activation of pyroptosis signaling pathway [6,7]. Activated NLRP3 may recruit and activate the precursor caspase 1, and inflammatory stimuli can boost NLRP3 transcription and activity. By activating caspase 1 of the inflammasome component, activation and assembly of the inflammasome enhance maturation, proteolytic cleavage, and release of pro-inflammatory cytokines such as interleukin (IL)-1(IL-1) and interleukin (IL)-18 (IL-18) [8]. The activated caspase cleaves and activates pore-forming effector protein Gasdermin D (GSDMD). GSDMD will cause pyroptosis by punching holes in the cell membrane and releasing pro-inflammatory cytokines such IL-1 a. The main clinicopathological type of AKI is renal tubular necrosis [9]. Pyroptosis of glomerular epithelial cells [10,11] and proximal renal tubular cells [12,13] is related to renal tubular necrosis.

The increased expression of NLRP3 under inflammation plays an important role in the subsequent activation of signal molecules and the mechanism of cell pyroptosis [14]. However, the molecular mechanism of inflammatory induced elevated NLRP3 expression to cell pyroptosis in renal tubular epithelial cell injury in septic-associated AKI is not clear. Furthermore, there has been no study on the upstream molecular mechanism of the increased expression of NLRP3.

In this study, it is hypothesized that cell pyroptosis caused by increased NLRP3 transcription levels after inflammatory stimulation is involved in the pathogenesis of AKI. In view of the reasons for the increase of NLRP3, the specific transcription factor was identified by analyzing the upstream promoter of NLRP3. Whether the transcription factor could affect cell pyroptosis and participate in the pathogenesis of AKI was also verified by regulating the transcription of NLRP3 to provide a molecular basis for inhibiting cell pyrophosphate and reducing kidney injury.

## Materials and methods

### 1. Patient data collection

Patients with AKI hospitalized at Second Affiliated Hospital of Soochow University from February 2020 to February 2021 were included. The health people in the control group were recruited from a healthy population who underwent health examination at the Second Affiliated Hospital of Soochow University from February 2020 to February 2021. Demographics, diagnostic codes (International Classification of Diseases 9/10 Clinical Modification [ICD-9/10-CM]), clinical data, and laboratory measurements of patients during the hospitalization were collected. The Second Affiliated Hospital of Soochow University’s Institutional Review Board approved the research protocol (ethic numbers: JD-LK-2021-003-01), and all patients gave their informed consent before treatment.

### 2. Cell culture

The American Type Culture Collection (ATCC, Manassas, VA, USA) provided human embryonic kidney (HEK) 293 cells and renal tubular epithelial cells (HK2), which were incubated in a complete DMEM medium at 37°C with 5% CO2. HEK293 cells and HK2 cells were stimulated with different concentrations of lipopolysaccharide (LPS, #L2880, Sigma-Aldrich, St. Louis, MO, USA) (0.1 μg/ml, 1 μg/ml, and 10 μg/ml) for 6 hours, 12 hours, and 24 hours, respectively, to imitate inflammation, and then treated with phosphate-buffered saline (PBS) as a control [15].

### 3. Enzyme-linked immunosorbent assay

TNF-α(#DTA00D), IL-18 (#DL180), and IL-1β (#DLB50) concentrations in the culture medium and serum were determined using commercial Enzyme-linked immunosorbent assay (ELISA) kits (R&D Systems, Minneapolis, MN, USA) according to the manufacturer’s instructions. Briefly, the ELISA was carried out according to the sandwich principles. The wells were pre-coated with antigen, and specific antibodies of the sample binding to the antigen-coated wells were detected by the secondary enzyme-conjugated antibody specific for human IgG. After a tetramethylbenzidine (TMB) substrate reaction, the intensity of the blue coloration was proportional to the quantity of detected IgG-specific antibodies. An automatic microplate reader read the optical density (OD) of the well at 450 nm with an automatic microplate reader [16]. According to the manufacturer’s guidelines, antibody activities were calculated using a standard curve.

### 4. *Construction of human NLRP3 promoter pGL3 luciferase reporte*r plasmid*s*

A 2046 bp fragment of human NLRP3 promoter was amplified and then inserted into upstream of pGL3-Basic vector (#E1751, Promega, Wisconsin, Madison, WI, USA) with the restriction enzyme Mlu I and Xho I. During this process, the forward and reverse primers used were 5′-CGACGCGTGTGATCCTCCTGCCTCAG-3′ (restriction site for Mlu I underlined) and 5′-CCGCTCGAGGGACAAGTTCTGCCCTCT-3′ (restriction site for Xho I underlined), respectively. To construct clones with different deletions of the 5′ end of the NLRP3 promoter region, various amplicons were produced according to the corresponding Mlu I sites [17]. The identical reverse primer and the forward primers for amplicons were as follows:

(−1216 to +100: 5′- CGACGCGT CTCCCAGGTTCAAGTGAT −3′);

(−798 to +100: 5′- CGACGCGT TGCAGTATAATGAAGGGATC −3′);

(−342 to +100: 5′- CGACGCGT TGAGTCAATGAGTCAGGGAG −3′);

(−257 to +100: 5′- CGACGCGT TCCCACCCTGCTTCTGTG −3′);

(−146 to +100: 5′- CGACGCGT GCCTCTGCTCTGATGTAAG −3′);

These sequences were confirmed using DNA sequence analysis. Then, these fragments were inserted into pGL3-Basic vector as mentioned above.

### 5. Plasmids and siRNAs

The promoter fragments of the ETS Proto-Oncogene 1 (ETS1) gene were amplified and inserted upstream of the pGL3-Basic vector (Promega, Wisconsin, USA) with the restriction enzymes Mlu I and Xho I. The plasmid pENTER-ETS1 for ETS1 overexpression and control vector pENTER were obtained from Verzen Biotechnology (#pAD100001-OE, Shandong, China). Genepharma (Shanghai, China) developed and produced a small-interfering RNA (siRNA) that targeted ETS1 and a non-target control siRNA. The ETS1 mRNA was targeted by siRNA, and the control sequence was presented below:

siETS1: 5′-GCAGCCAGUCAUCUUUCAATT-3′

control: 5′-UUCUCCGAACGUGUCACGUTT-3′

### 6. Site-directed mutagenesis

The QuikChange Site-Directed Mutagenesis kit (#R401, Takara Ltd., Otsu, Japan) was used to create mutations in the transcriptional factors’ specific binding sites in the NLRP3 promoter region. After mutation, the sequences were further confirmed by the DNA sequencing analysis [18].

### 7. Transient transfections and dual-luciferase reporter assays

HEK293 and HK2 cells were plated into 96-well plates 24 hours before transfection. Cells were co-transfected with 400 ng of various luciferase plasmids and 4 ng of pRL-TK plasmid (#16154, Invitrogen, Carlsbad, CA, USA) using Lipofectamine-3000 transfection reagent (#L3000015, Invitrogen, Carlsbad, CA, USA). After 48 hours of transfection, the luminescence was measured by the TD-20/20 luminometer (Turner Designs, Sunnyvale, USA) in a dual reporter assay system (Promega, Wisconsin, USA). The results were derived from at least three separate experiments, each of which was performed in triplicate wells. Overexpression plasmids (300 ng) or siRNA (50 nM) were co-transfected with NLRP3 promoter reporter plasmids (100 ng) into HEK 293 cells under overexpression or RNA interference conditions, respectively. The co-transfection was followed by a 48-hour luciferase test [17].

### 8. Chromatin immunoprecipitation assay

In this experiment, the Magna ChIP TM kit (#17e611, Millipore, Billerica, MA, USA) was used following the manufacturer’s instructions. Additionally, 1χ10^7^ HK2 cells were incubated in 1% formaldehyde at room temperature for 10 min. Cells were then washed thoroughly with ice-cold PBS before being collected by centrifugation at 4°C for 10 min. On a sonicator ultrasonic processor, the cell pellets were re-suspended in roughly 500 l nuclear lysis buffer and sonicated using six 15 sec pulses with a 50-second break throughout the pulse interval at 5% of maximum output intensity (#Q800R, Qsonica LLC, Newtown, CT, USA). Anti-ETS1 ChIP level antibody (#ab225868, Abcam, Eugene, OR, USA) and rabbit IgG control antibody (#sc-2027, Santa Cruz Biotechnology, CA, USA, USA) were used to precipitate ultrasonically fragmented chromatin fragments (Millipore). Quantitative PCR (Q-PCR) was used to amplify the precipitated and purified DNA using ABI 7300 real-time PCR equipment (Applied Biosystems Inc, Foster City, CA, USA) [18]. Primers were forward 5′- CGAGACACGGTTTTGACA −3′ and reverse 5′- ACACTGCCCCGCGGAGCT-3′ .

### 9. RNA extraction and real-time Q-PCR

TTRIzol reagent was used to extract the total RNA of the cells. After Chloroform extraction and isopropanol precipitation, cells were washed with 75% ethanol. The RNA was then reverse transcribed into cDNA using RNA reverse transcriptase (#RR036A, Takara Ltd., Otsu, Japan). For real-time quantification of gene transcripts, TB Green Premix Ex Taq II (#RR820A, Takara Ltd., Otsu, Japan) and ABI 7300 real-time PCR equipment from Applied Biosystems Inc. were adopted. In addition, GAPDH was used as an internal reference. Primer sequences were as follows:

NLRP3:

F: 5’-GATGGGTCAAGATGGCATCG-3’

R: 5’-AAGTTCTCCTGTTGGCTCGA-3’

ETS1:

F: 5’-TAAGTGAGGTGCTGAGAGCG-3’

R: 5’-CCCAAAAGGGGTAGCAAGGT-3’

GAPDH:

F: 5’-CGGAGTCAACGGATTTGGTCGTAT-3’

R: 5’-AGCCTTCTCCATGGTGGTGAAGAC-3’

### 10. Western blot analysis

All collected cells were lysed in Laemmli buffer, and the released cell proteins were boiled to denature. Then, the western blot was performed as previously described. Briefly, equal amounts of protein were separated by sodium dodecyl sulfate (SDS)-polyacrylamide gel electrophoresis and then transferred to a polyvinylidene difluoride membrane. The membrane was incubated overnight with corresponding primary antibodies. Antibodies against NLRP3 (#ab263899), Gasdermin D (#ab210070), and GAPDH (#ab8245) were purchased from Abcam (Cambridge, UK), and those against cleaved Caspase 1 (#89332) was purchased from Cell Signaling Technology (Danvers, MA, USA). Peroxidase-conjugated IgG (#SA00001-2, Proteintech, Wuhan, China) was used as a secondary antibody. Finally, bands were quantified by densitometry using ImageJ software.

### 11. Cell proliferation assay

HK2 cells were planted at a density of 1.0χ10^3^/well in 96-well plates. Before detection, the culture medium was evacuated, and cells were stained with Cell Counting Kit-8 (CCK-8 kit, #CK04, Dojindo, Kumamoto, Japan). Thermo Scientific Multiskan FC (ThermoFisher, Waltham, MA, USA) was used to measure the absorbance at 450 nm after 1 hour of incubation at 37°C (Waltham, MA, USA). The following formula was used to calculate cell proliferation activity: proliferation activity (%) = [A (delivery) – A (blank)]/[A (control) – A (blank)] multiplied by 100.

### 12. Electrophoretic mobility shift assay (EMSA)

EMSA was performed using the Gel Shift Kit (#E3300, Promega, Madison, WI, USA). For EMSA, Wt and Mut short oligonucleotide probes were synthesized by GenePharma (Shanghai, China). A typical binding reaction was conducted by incubating the purified ETS1 protein with a biotin-labeled DNA probe at room temperature for 20 min. The binding products were then resolved on an 8% polyacrylamide gel in 0.5 X Tris-borate-EDTA. For the super-shift assay, 2 μg of the anti-ETS1 antibody was added to the nuclear extracts. Finally, signal intensities of bands on the gel were visualized using the ChemiDoc MP Imaging System (BIO-RAD) [18]. The sequences of probes were as follows:

Wt: forward 5’-GTGGAGACCACATCCTTCCTGCCCCTTCTGGGGCTGCGAC-3’

Wt: reverse 5’- GTCGCAGCCCCAGAAGGGGCAGGAAGGATGTGGTCTCCA-3’

Mut-forward 5’-GTGGAGACCACATCCTTCCTGCCCCTTCTGGGGCTGCGAC-3’

Mut-reverse 5’-GTCGCAGCCCCAGAAGGGGCAGGAAGGATGTGGTCTCCA-3’

### 13. Statistical analysis

The findings of this investigation were analyzed using SPSS 20.0 software (SPSS Inc., Chicago, IL, USA). The data were presented as the mean and standard deviation (SD). The paired t-test was used for intra-group comparisons conforming to normal distribution and chi-squaredness. Inter-group comparisons and multi-group comparisons were performed through the unpaired t-test and the one-way ANOVA, respectively. The LSD-test was used for two-group comparisons, and the rank-sum test was used for data that did not conform to normal distribution and chi-squaredness. A significant difference was defined as a *P* value less than 0.05.

## Results

In this study, we identified the inflammatory state and pyroptosis level in AKI patients. A series of studies were conducted to explore the transcriptional mechanism of up-regulated expression of NLRP3, an essential gene leading to cell pyroptosis, and to provide a novel molecular theoretical basis for the pathogenesis of AKI.

### 1. Inflammatory cytokines and NLRP3 were elevated in AKI patients and LPS-treated renal tubular epithelial cells

In order to explore the levels of inflammatory cytokines and NLRP3 expression in AKI patients, peripheral blood samples from patients and healthy controls were collected for detection (Table 1). The levels of cytokines TNF-α, IL-18, and IL-1β in peripheral blood serum were detected by ELISA, and the expression level of NLRP3 was detected by qPCR. The results showed that TNF-α, IL-18, and IL-1β levels were significantly higher in AKI patients than healthy controls (Figure 1(a), **P < 0.01, ***P < 0.001). The expression level of NLRP3 was also significantly higher than that of healthy controls (Figure 1(b), **P < 0.01).

**Figure 1.** **Levels of inflammatory cytokines and NLRP3 were elevated in patients with AKI.** (a) The levels of cytokines TNF-α, IL-18 and IL-1β in serum of peripheral blood were detected by ELISA. (b) The expression level of NLRP3 in AKI patients was detected by qPCR. (**P<0.01, ***P<0.001).

**Table 1.** Clinical data of AKI patients and normal controls

Factors	AKI patients	Normal controls
Over all (n)	54	43
Gender (n)		
Male	36	25
Female	18	18
Age (year)	52.6 ± 6.8	55.9 ± 7.6
Etiological Factor (n (%))		
Prerenal factors	7 (13.0)	–
Renal factors	42 (77.8)	–
Nephrotic syndrome	28 (51.9)	–
Infection	6 (11.1)	–
Drugs	4 (7.4)	–
The others	4 (7.4)	–
Postrenal factors	5 (9.2)	–

In order to simulate the effect of infection status on the NLRP3 expression level and cell pyrolysis, we stimulated different cell lines (HEK cells, HEK293 and Human Kidney-2, HK2) with varying concentrations of LPS (PBS, 0.1 μg/ml, 1 μg/ml, and 10 μg/ml) for different time (0 h, 6 h, 12 h, and 24 h), and detected the NLRP3 transcription level by qPCR. The results showed that in HEK293 cells (Figure 1(c)), 1 μg/ml LPS for 12 h resulted in a significant increase in NLRP3 mRNA expression (F = 107.6, ***P < 0.001). The expression level of NLRP3 in HK2 cells (Figure 1(c)) showed the same trend after LPS stimulation, but its increase was more significant (F = 100.7, ***P < 0.001).

It has been reported that NLRP3 inflammasome is a crucial factor in inflammation and can promote pyroptosis [19]. The effect of the up-regulated expression level of NLRP3 on pyroptosis was further investigated by detecting cell viability and key molecular levels of pyroptosis. The cell viability was lower in the LPS-treated group than in the control group (Figure 1(d)). Additionally, the concentrations of IL-18 and IL-1β (Figure 1(e)) and the levels of pyroptosis-related proteins (Figure 1(f)) were higher in HK2 cells exposed to LPS than in PBS. Hence, it is concluded that LPS can increase the NLRP3 level and aggravate pyroptosis of HK2 cells.

### 2. Identification of the human NLRP3 gene transcription start site (TSS) and the core region of the human NLRP3 gene promoter

Based on the above results, we found that the increased NLRP3 expression level can lead to alterations in HK2 pyroptosis and may be involved in AKI. Thus, we intended to further study the transcriptional regulation mechanism of the NLRP3 gene. To identify the human NLRP3 gene promoter, we employed DBTSS Program (https://dbtss.hgc.jp/) to search potential sequences. For the efficiency of the dual-luciferase reporter gene, HEK293 cells with high transfection efficiency were selected. It revealed the presence of a putative promoter at nucleotides −250 in the HEK293 5ʹflanking region (Figure 2(a)). The human NLRP3 gene promoter region includes multiple potential transcription factor-binding sites, such as ETS1, VDR, SPI1, and ALX3, according to sequence analysis using UCSC software (http://genome.ucsc.edu/) (Figure 2(b)).

**Figure 2.** **LPS up-regulated NLRP3 in renal tubular epithelial cells and promoted cell pyroptosis.** (a) NLRP3 mRNA expression level was observed after different concentrations of LPS treatment for different time. (b) The cell viability was evaluated after LPS or PBS treatment by CCK-8 assay. (c) The levels of cytokines TNF-α, IL-18 and IL-1β were detected by ELISA in LPS or PBS treated HK2 cells. (d) The pyroptosis-related proteins’ levels were detected by WB. (**P<0.01, ***P<0.001).

In order to further determine the regulatory elements of the NLRP3 gene, the 2046 bp (relative to TSS-1946 to +100) fragment of the promoter region predicted by the software was cloned into the promoter-free pGL3-basic luciferase reporter plasmid and defined as pGL-1946. Then, HEK293 cells were transiently transfected using plasmid pGL-1946. It produced a substantial luciferase activity in HEK293 cells (35 times more than PGL3-BASIC), suggesting that it includes the human NLRP3 promoter region, as shown in (Figure 2(c)). The whole 2046 bp portion of the human NLRP3 promoter region was shortened into several sections before being placed into the PGL3-Basic vector and then transfected to determine promoter activity and discover the minimal promoter sequence responsible for human NLRP3 gene transcription. The +100 bp location (relative to TSS) was constant at the 3’ end of these promoters but was varied at the 5’ end. The promoter activity of pGL3 + 18 was low, according to luciferase tests. The promoter activities of pGL3-1946, −1216, −798, −342, −257, and −146 were significantly high (Figure 2(c, f) = 80.44, ***P < 0.001). These findings suggest that sequences between −146 and +18 are adequate for inducing NLRP3 basal transcription.

### 3. Functional analysis of putative binding sites for ETS1 in the human NLRP3 gene promoter

Through online software (TFSEARCH, UCSC), we predicted the binding sites of transcription factors in the minimum promoter active region (−146bp ~ +18bp). Several speculated binding sites, including ETS1, VDR, SPI1, and ALX3, were found in this region (Figure 3(a)). The specific sequence of binding sites is shown in (Figure 4(a)). To assess the effect of putative binding sites on transcriptional regulation of NLRP3 promoters, site-directed mutagenesis was performed on key bases of these putative binding sites and then reporter plasmids were inserted (Figure 3(b)). Promoter activity of mutant and wild-type plasmids was analyzed. As shown in (Figure 3(c)), ETS1 point mutation resulted in the most significant decrease of NLRP3 promoter activity (15% of the wild-type promoter activity). The activity of the SPI1 mutant plasmid promoter was 88% of that of the wild-type promoter (* *P = *0.0475). The activity of the VDR or ALX3 mutant plasmid promoters was comparable to that of the wild-type promoter (Figure 3(c)). These results indicated the most important role of the ETS1 site in basal transcription of NLRP3.

**Figure 3.** **Identification of the human NLRP3 gene transcription start site (TSS) and promoter region core region in the human NLRP3 gene promoter.** (a) The promoter region and transcription initiation site of NLRP3 gene predicted by the DBTSS Program. (b) NLRP3 promoter analyzed via UCSC Genome Browser and ETS1predicted as the transcription factor of NLRP3 gene. (c) The human NLRP3 promoter sequence with different 5′ end (from −1946/+100 to +18/+100) was ligated to the firefly luciferase and inserted into plasmid pGL3 basic. (*** *P* < 0.001).

**Figure 4.** **Functional analysis of putative binding site for ETS1 in human NLRP3 gene promoter.** (a) Detailed information of NLRP3 promoter’s motifs. (B) Point mutationsof putative binding sites. (c) Mutation analysis of the transcription factors binding sitesin the human NLRP3 promoter. (d) ETS1 knockdown and overexpression efficiency were confirmed by RT-qPCR analysis. (e) The expression level of NLRP3 mRNA was detected after the knockdown or overexpression of ETS1. (f) Relative luciferase activity of the NLRP3 promoter was detected cells by cotransfected with ETS1overexpression vectors pENTER-ETS1 (plasmids pENTER as the control), siRNAinterference siETS1(negative control siRNA as the control) and NLRP3 reporter plasmids together with renilla luciferase plasmid pRL-TK into HEK293 cells. (**P<0.01, *** *P* < 0.001).

The transcription factor ETS1 was overexpressed and knocked down to establish the ETS1 site as a crucial regulator. RT-qPCR research validated the effectiveness of siRNA directed against ETS1 and the overexpressed plasmid on ETS1 mRNA levels (Figure 3(d)). With the knockdown or overexpression of ETS1, the expression level of NLRP3 mRNA was down-regulated or up-regulated (Figure 3(e)).

In addition, ETS1 overexpression was found to boost the activity of the NLRP3 promoter by 1.7 times (Figure 3(f)). We employed RNA interference to knock down ETS1 expression in HEK293 cells to validate its control on NLRP3 promoter activity. In HEK293 cells, we cotransfected the NLRP3 reporter plasmid with ETS1 siRNA or a negative control siRNA. The presence of ETS1-specific siRNA resulted in a 63% decrease in luciferase activity compared to the negative control siRNA (Figure 3(f)).

We inferred that ETS1 positively regulated the baseline transcriptional activity of NLRP3 based on the aforementioned experimental findings.

### 4. Binding of ETS1 to NLRP3 promoter region in HK2 cells

EMSA and ChIP assays were performed to observe whether ETS1 exerted a direct or indirect influence on NLRP3 expression. DNA-protein complexes were formed between the labeled ETS1-binding oligonucleotide probe and the nuclear protein in cells from the HK2 cell line, as shown in (Figure 4(a)). (lane 2). Utilizing a competitive probe with extra unlabeled material and a mutant probe, the specificity of the ETS1-DNA interaction was confirmed (lanes 3 and 4). Moreover, an anti-ETS1 antibody was employed to conduct super-shift assays. As shown in (Figure 4(a)), the addition of an anti-ETS1 antibody resulted in a decrease in the number of specific complexes (lane 5), indicating the specific binding of ETS1 to the NLRP3 promoter. To demonstrate the binding of ETS1 to the NLRP3 promoter in vivo, we conducted ChIP on LPS-treated HK2 cell extracts using an anti-NLRP3 antibody. The ETS1-relevant chromatin fragments were immunoprecipitated with specific ETS1 antibodies, and the purified DNA product served as a template. Primers around the potential binding site of ETS1 were designed for the active region of the NLRP3 gene promoter, and real-time Q-PCR was performed to amplify the DNA fragment. (Figure 4b)) showed that the ETS1 antibody was specifically bound to the amplified sequence of the NLRP3 promoter region in vivo by immunoprecipitation. Moreover, the binding ability of ETS1 and NLRP3 was significantly enhanced after LPS treatment. The bar chart below showed the quantification of chromatin fragments by Q-PCR. The comparison of the ETS1 antibody and a nonspecific IgG control antibody revealed a substantial enrichment of the NLRP3 promoter (Figure 4(b)).

These data suggested that ETS1 could bind to the NLRP3 promoter region in vivo and vitro.

### 5. Alleviation of the pyroptosis of renal tubular epithelial cells through NLRP3 transcription regulation by knocking down ETS1

The above experiments indicated that ETS1 up-regulated NLRP3 by binding to the transcription site of NLRP3. Q-PCR revealed that ETS1 mRNA expression was significantly elevated in the peripheral blood of AKI patients compared with that in controls (Figure 5(a), **P = 0.0036). Given that LPS could up-regulate the expression of NLRP3 in renal tubular epithelial cells and promote cell pyroptosis, we will next explore the transcriptional mechanism of NLRP3 up-regulation and the promotion mechanism of cell pyroptosis after LPS treatment.

**Figure 5.** **ETS1 specifically binds to the promoter of NLRP3 as shown by EMSA and ChIP analyses.** (a) (EMSA analysis) Nuclear extracts were prepared from HK2 cells and used for EMSA analysis. (b) (ChIP analysis) A representative gel image of PCRproducts obtained from ChIP of HK2 cells. (**P< 0.01).

First, the expression levels of ETS1 mRNA (Figure 5(b)) and protein (Figure 5(c)) were elevated (***P < 0.001) in LPS-treated HK2 cells. We found that the expression level of ETS1 increased after LPS treatment, positively correlated with that of NLRP3 (Figure 5 (d), r = 0.9135, ***P < 0.001). Subsequently, we used siRNA interference technology to knock down ETS1, which was found to reverse the cell viability (Figure 5 (e, f) = 112.7, ***P < 0.001) and reduce the upregulated levels of NLRP3 and cell pyroptosis after LPS treatment (Figure 5(f)).

Thus, we concluded that ETS1 participated in the AKI pathogenesis by regulating the transcription of NLRP3 and affecting the pyroptosis of renal tubular epithelial cells.

## Discussion

AKI is a major healthcare challenge worldwide [20] and is induced by a variety of factors, among which pathogen infection is the most common [21]. Consistent with previous clinical reports [22,23], we also noted that infection was an important pathogenic factor of AKI in the collected cases. Inflammation can change cellular biological behavior. Sepsis mediates apoptosis through endoplasmic reticulum stress in renal tubular cells [24]. Proximal renal tubular necrosis in AKI is defined by injury or death of renal tubular epithelial cells [25,26], and the role of pyroptosis in AKI has been proven. TLR4/NF-κB is a classic LPS-induced inflammatory signaling pathway. After microbial infection, NLRP3 inflammasome is activated through TLR4/NF-κB pathway with an increased expression level, acting as an important molecule in cell pyroptosis [27,28]. α-Klotho protein has a therapeutic activity in contrast-induced AKI by limiting NLRP3 inflammasome-mediated pyroptosis [29]. The increased NLRP3 expression and pyroptosis level in AKI patients indicated LPS-induced NLRP3-dependent pyroptosis in AKI., consistent with previous results [30,31].

The increased expression of NLRP3 is an important link in the pathogenesis of cell pyroptosis [32,33] and AKI [34,35], and thus its mechanism should be explored. In eukaryotic cells, gene expression changes are mainly caused by cis-regulation of the upstream promoter transcription factor [36,37]. The transcriptional regulation mechanism of NLRP3 expression elevation after exogenous infection stimulation remains unclear. ETS-1 is a transcription factor, responsible for regulating the expression of a variety of genes, including growth factors, chemokines, and adhesion molecules [38]. The renal expression of ETS-1 increases in various models of renal injury [39,40]. External environmental stimuli can affect the transcriptional activity of ETS1, thus preventing its binding ability with downstream target genes. For example, calmodulin-dependent kinase II can inhibit the activity of ETS1 and its binding to DNA by preventing threonine phosphorylation [41,42]. In addition, the expression level of ETS1 is directly up-regulated to control the transcription of target genes [43]. For example, after LPS or TNF-α stimulation, the expression level of ETS1 increases and depends on the expression level of NF-κB [44]. Our study highlights ETS1 expression changes can affect NLRP3 expression and cell pyroptosis. Previous studies have also shown that ETS1 can promote apoptosis [45,46]. To our knowledge, the present study, for the first time, identified the upstream transcription factor ETS1 of NLRP3 and further refined the mechanism of ETS1 promoting cell death.

In addition, ETS1 is a mediator that promotes kidney inflammation and fibrosis [47] and leads to kidney injury by damaging cell endothelium [48]. ETS1 plays an important role in diabetic nephropathy and hypertensive nephropathy-related renal damage. Our study confirmed the promoting role of ETS1 in the pathogenesis of sepsis-associated AKI. In LPS-induced renal tubular epithelial cell injury, down-regulation of ETS1 alleviated pyroptosis, suggesting ETS1 as a potential target for AKI treatment.

## Conclusion

Our data demonstrate that in the pathogenesis of AKI, ETS1 can activate NLRP3 promoter activity through the upstream transcription site of NLRP3 promoter, increase NLRP3 expression and promote pyroptosis of renal tubular epithelial cells. Therefore, this study will provide a new understanding of the link between transcription factors ETS1 and NLRP3 and lay a molecular basis for targeted treatment of AKI.

## Supplementary Material

Supplemental Material
